# Prognostic significance of metastatic lymph node ratio in gastric cancer: ﻿a Western-center analysis

**DOI:** 10.1186/s12893-023-02127-y

**Published:** 2023-08-07

**Authors:** Muhammer Ergenç, Tevfik Kıvılcım Uprak, Muhammed İkbal Akın, Ece Elif Hekimoğlu, Çiğdem Ataizi Çelikel, Cumhur Yeğen

**Affiliations:** 1 Department of General Surgery, Marmara University School of Medicine, Başıbüyük Campus Başıbüyük Mah. Maltepe Başıbüyük Yolu Sok. No: 9/1 Maltepe 34854, Istanbul, Turkey; 2 Marmara University School of Medicine, Başıbüyük Campus Başıbüyük Mah. Maltepe Başıbüyük Yolu Sok. No: 9/1 Maltepe 34854, Istanbul, Turkey; 3 Department of Pathology, Marmara University School of Medicine, Başıbüyük Campus Başıbüyük Mah. Maltepe Başıbüyük Yolu Sok. No: 9/1 Maltepe 34854, Istanbul, Turkey

**Keywords:** Gastrectomy, Lymph node ratio, Metastatic lymph node ratio, Survival, Prognosis

## Abstract

**Background:**

Tumor-node-metastasis (TNM) staging is the central gastric cancer (GC) staging system, but it has some disadvantages. However, the lymph node ratio (LNR) can be used regardless of the type of lymphadenectomy and is considered an important prognostic factor. This study aimed to evaluate the relationship between LNR and survival in patients who underwent curative GC surgery.

**Methods:**

All patients who underwent radical gastric surgery between January 2014 and June 2022 were retrospectively evaluated. Clinicopathological features of tumors, TNM stage, and survival rates were analyzed. LNR was defined as the ratio between metastatic lymph nodes and total lymph nodes removed. The LNR groups were classified as follows: LNR0 = 0, 0.01 < LNR1 ≤ 0.1, 0.1 < LNR2 ≤ 0.25 and LNR3 > 0.25. Tumor characteristics and overall survival (OS) of the patients were compared between LNR groups.

**Results:**

After exclusion, 333 patients were analyzed. The mean age was 62 ± 14 years. According to the LNR classification, no difference was found between groups regarding age and sex. However, TNM stage III disease was significantly more common in LNR3 patients. Most patients (43.2%, *n* = 144) were in the LNR3 group. In terms of tumor characteristics (lymphatic, vascular, and perineural invasion), the LNR3 group had significantly poorer prognostic factors. The Cox regression model defined LNR3, TNM stage II—III disease, and advanced age as independent risk factors for survival. Patients with LNR3 demonstrated the lowest 5-year OS rate (35.7%) (estimated mean survival was 30 ± 1.9 months) compared to LNR 0–1–2.

**Conclusion:**

Our study showed that a high LNR was significantly associated with poor OS in patients who underwent curative gastrectomy. LNR can be used as an independent prognostic predictor in GC patients.

## Background

One of the most prevalent malignancies in the world and the fourth-leading cause of cancer-related mortality is gastric cancer (GC). GC is a typical sample of neoplasia that evolves against a background of chronically inflamed mucosa, and risk factors include multiple variables that cannot be modified, such as age, gender, and race/ethnicity. Controllable risk factors comprise infection with Helicobacter pylori bacteria, smoking, and diets high in nitrates and nitrites. New prognostic and/or therapeutic tumor markers are needed to improve poor survival outcomes and aid early cancer detection. However, there are no perfect markers specific to GC. With a better understanding of the mechanisms underlying gastric carcinogenesis, numerous molecular targets have been identified that can be used as biomarkers with diagnostic and prognostic potential. The use of novel biomarkers in the early detection of GC could reduce mortality and medical costs. Preoperative sCD26 levels may be a useful and easy biomarker for the early diagnosis of GC [1–6].

Surgical resection is the main curative therapy for stomach cancer, and lymph node metastasis is a prognostic indicator. Thus, lymph node status is crucial in postoperative survival in GC [7, 8]. The primary staging method for GC is tumor-node-metastasis (TNM) staging. This approach bases the node factor on the number of positive lymph nodes, and the D1, D2, and D3 lymph node dissection levels impact the N stage. The N stage should be correctly determined by examining at least 15 lymph nodes. However, the surgeon's specialization, the experience of the pathologist, and other inevitable circumstances might lead to analyzing fewer than 15 lymph nodes, resulting in "stage migration". Hence, patients with insufficient lymphadenectomy receive an inaccurate prognosis evaluation based on their TNM stage [7, 9–13].

Exact staging in the TNM method may not be guaranteed by D1 lymph node dissection restricted to the perigastric lymph nodes. However, the lymph node ratio (LNR), which is regarded as a significant prognostic indicator and a suitable staging approach for patients with positive lymph nodes, can be utilized independently of the type of lymphadenectomy. Studies comprising extensive case series have demonstrated that LNR may reliably determine the prognosis of GC patients further than node stage [7, 9, 10, 14].

In this study, we aimed to assess the correlation between LNR and survival in patients who underwent curative GC surgery.

## Methods

Patients diagnosed with gastric adenocarcinoma after radical gastric surgery at Marmara University Hospital between January 2014 and June 2022 were retrospectively examined.

The Marmara School of Medicine Clinical Research Ethics Committee approved this research with number 08.10.2022.1081.

Patients diagnosed with gastric adenocarcinoma by histopathologic examination, patients who underwent R0 resection and D1 and D2 lymphadenectomy, and patients with complete follow-up data were included [15, 16]. Patients with a history of cancerous tumors at other locations or gastric stump cancer, patients with a preoperative or operative distant metastasis diagnosis, multivisceral resections, esophageal cancer, and those who underwent neoadjuvant treatment were excluded from the study. By excluding patients who had 15 or fewer nodes removed, we aimed to lessen the effects of varying surgical quality [17].

Age, sex, comorbidities, operation type, TNM stage, tumor sites, pathological features, and classification of tumors were examined.

Based on the number of metastatic lymph nodes, lymph node status was classified according to the seventh edition of the UICC/AJCC tumor-node-metastasis system [18]. LNR was defined as the ratio between metastatic lymph nodes and total lymph nodes removed. LNR ranged from 0 to 1 and was stratified based on previous studies; it was used to compare overall survival (OS) within each interval and between bordering subgroups with similar survival outcomes. The LNR groups were classified as follows: LNR0 = 0, 0.01 < LNR1 ≤ 0.1, 0.1 < LNR2 ≤ 0.25 and LNR3 > 0.25 [19, 20].

The primary outcome of this study was to determine the effect of the LNR on OS. The secondary outcome was to identify other factors that impact OS.

### Statistical analysis

We used the Statistical Package for Social Sciences (Version 25.0. Armonk, NY: IBM Corp.) for our statistics. We assessed the distribution of continuous data for normality using the Kolmogorov‒Smirnov and Shapiro‒Wilk normality tests. A log-rank test was performed to evaluate significant differences between groups, and we computed the OS rate using the life table approach. Survival curves were used using the Kaplan‒Meier method. The multivariate Cox proportional hazards model included each parameter from the univariate analysis that passed statistical thresholds for significance. We used the area under the curve (AUC) and receiver operating characteristic (ROC) curvilinear analyses to examine the predictive evaluation accuracy of various staging systems. We considered a *p*-value of less than 0.05 to indicate statistical significance.

## Results

Between January 2014 and June 2022, 776 patients operated on at Marmara University Hospital for GC were analyzed retrospectively. Twenty patients were excluded from the research because the T value was unknown, and eight patients were excluded because the N value was unknown. Twelve patients underwent completion gastrectomy, 11 patients underwent Ivor Lewis, and 16 patients whose surgical information could not be reached were excluded from the study. Two hundred fifty-four patients were excluded because fewer than 16 lymph nodes were removed, and 80 patients received neoadjuvant therapy (Fig. 1).

**Fig. 1:** Flowchart of patient selection

Excluding patients removed from the study, of the remaining 333 patients, 103 (30.9%) were female, and 230 (69.1%) were male. The patients' ages ranged from 19 to 90 years old, with a mean age of 62 ± 12.

Tumors were observed in four different regions according to stomach localization. Of these regions, 111 (33.3%) were in the distal 1/3, 73 (21.9%) were in the cardia, 116 (34.9%) were in the corpus, and 33 (9.9%) were in the linitis plastica. Detailed perioperative clinical features of the patients are given in Table 1.

**Table 1:** Patients’ demographics and perioperative clinical characteristics

Parameters		*N* = 333	%
**Age (years, mean ± SD)**		62 ± 12	
**Sex**	Male	230	69.1%
	Female	103	30.9%
**Tumor-node-metastasis (TNM) Stage**	I	42	12.6%
	II	62	18.6%
	III	229	68.8%
**Operation type**	Total gastrectomy	152	45.6%
	Subtotal gastrectomy	158	47.5%
	Proximal gastrectomy	23	6.9%
**Tumor site**	Upper third	73	21.9%
	Middle third	116	34.9%
	Lower third	111	33.3%
	Linitis Plastica	33	9.9%
**World Health Organization (WHO) classification**	Tubular	63	18.9%
	Solid	8	2.4%
	Poorly cohesive	51	15.3%
	Mixed	207	62.2%
	Unknown	4	1.2%
**Lauren classification**	Intestinal type	176	52.9%
	Diffuse type	57	17.1%
	Mixed	100	30%
**Tumor size (cm, median—range)**		5.5 (1—20)	
**Lymphatic invasion**	Absent	47	14.1%
	Present	286	85.9%
**Vascular invasion**	Absent	141	42.3%
	Present	192	57.7%
**Perineural invasion**	Absent	88	26.4%
	Present	245	73.6%
**Lymph Node Ratio (LNR)**	LNR0	75	22.5%
	LNR1	55	16.5%
	LNR2	59	17.7%
	LNR3	144	43.3%

Total gastrectomy was performed in 152 (45.6%) patients, subtotal gastrectomy in 158 (47.5%) patients, and proximal gastrectomy in 23 (6.9%) patients. While intestinal-type tumors were observed in the majority of patients (52.9%), mixed-type tumors (62.2%) were also mainly detected according to the WHO classification.

Patients were divided into four groups using the LNR classification system mentioned in the Methods section. Most patients (43.2%, *n* = 144) were in the LNR3 group. Considering the metastatic lymph node ratios, the mean value was 0.29, and the median value was 0.17 (0—1).

Age and sex differences between LNR groups were not observed. However, TNM stage III disease was significantly more common in LNR3 patients. In terms of tumor characteristics (lymphatic, vascular, and perineural invasion), the LNR3 group had significantly poorer prognostic factors (Table 2).

**Table 2:** Clinicopathological features according to lymph node ratio

Parameters		LNR0 *n* = 75 (%)	LNR1 *n* = 55 (%)	LNR2 *n* = 59 (%)	LNR3 *n* = 144 (%)	*P*-value
**Age (years, mean ± SD)**		64 ± 11	62 ± 12	60 ± 12	63 ± 12	0.241
**Sex**	Male	51 (68)	41 (74.5)	45 (76.3)	93 (64.6)	0.30
	Female	24 (32)	14 (25.5)	14 (23.7)	51 (35.4)	
**Tumor-node-metastasis (TNM) Stage**	I	38 (50.7)	2 (3.6)	1 (1.7)	1 (0.7)	** < 0.001**
	II	30 (40)	22 (40)	8 (13.6)	2 (1.4)	
	III	7 (9.3)	31 (56.4)	50 (84.7)	141 (97.9)	
**World Health Organization (WHO) classification**	Tubular	26 (34.7)	15 (27.3)	10 (16.9)	12 (8.3)	** < 0.001**
	Solid	3 (4)	3 (5.5)	0	2 (1.4)	
	Poorly cohesive	7 (9.3)	6 (10.9)	9 (15.3)	29 (20.1)	
	Mixed	38 (50.7)	31 (56.3)	40 (67.8)	98 (68.1)	
	Unknown	1 (1.3)	0	0	3 (2.1)	
**Lymphatic invasion**	Absent	35 (46.7)	6 (10.9)	2 (3.4)	4 (2.8)	** < 0.001**
	Present	40 (53.3)	49 (89.1)	57 (96.6)	140 (97.2)	
**Vascular invasion**	Absent	54 (72)	30 (54.5)	22 (37.3)	35 (24.3)	** < 0.001**
	Present	21 (28)	25 (45.5)	37 (62.7)	109 (75.7)	
**Perineural invasion**	Absent	46 (61.3)	18 (32.7)	8 (13.6)	16 (11.1)	** < 0.001**
	Present	29 (38.7)	37 (67.3)	51 (86.4)	128 (88.9)	

*LNR* Lymph node ratio

Univariable Cox regression analysis determined that TNM stage (hazard ratio (HR): 5.67; 95%-CI: 2.66–12.09, *p* < 0.001), lymphatic invasion (HR: 3.63; 95%-CI: 1.98–6.67, *p* < 0.001), perineural invasion (HR: 2.30; 95%-CI: 1.59–3.34, *p* < 0.001), age (HR: 1.03; 95%-CI: 1.02–1.04, *p* < 0.001), and LNR (HR: 2.72; 95%-CI: 1.97–3.77, *p* < 0.001) had a significant effect on overall survival.

The final multivariable Cox regression model defined LNR3, TNM stage II—III disease, and advanced age as independent risk factors for survival. At the same time, sex had no significant effect on overall survival (Table 3).

**Table 3:** Cox regression analysis of overall survival according to clinicopathologic factors

Parameters	Estimate	95% CI		Odds ratio	*P*-value
		**Lower**	**Upper**		
**LNR 0**	Ref -				
**LNR 1**	-0.1128	-1.0371	0.8115	0.893	0.811
**LNR 2**	-0.9199	-1.9124	0.0725	0.399	0.069
**LNR 3**	-1.3856	-2.3604	-0.4108	0.250	**0.005**
**TNM Stage I**	Ref -				
**TNM Stage II**	-1.4735	-2.6923	-0.2546	0.229	**0.018**
**TNM Stage III**	-1.6851	-2.9911	-0.3791	0.185	**0.011**
**Age (years)**	-0.0374	-0.0585	-0.0163	0.963	** < 0.001**
**Sex**					
Male	Ref -				
Female	0.0684	-0.4595	0.5963	1.071	0.800

*LNR* Lymph node ratio, *TNM* Tumor-node-metastasis

Overall, the 5-year survival was 52.7% in all patients. The median overall survival follow-up time was 26 months (range: 1–101 months). There was a significant difference in survival (*p* = 0.0001) between LNR groups (Fig. 2). Patients with LNR3 demonstrated the lowest 5-year OS rate (35.7%) (estimated mean survival was 30 ± 1.9 months) compared to LNR 0–1–2.

**Fig. 2:** Overall survival curve of the patients

## Discussion

According to extensive studies that have been conducted on prognostic variables for stomach cancer, the prognosis is generally thought to be related to clinicopathological factors (such as the location of the tumor, the depth of invasion, lymph node metastasis, and other factors) and treatment (such as surgery), in addition to lymph node dissection. The clinician may be able to more correctly evaluate the progression of the disease with the assistance of clinical and lymph node staging, as well as create a customized treatment plan that is complete and evaluates treatment and prognosis [7].

A study evaluating the quality of lymphadenectomy in GC has shown that extended lymphadenectomy (D2) is more predictive of disease-specific survival in GC patients, independent of the number of lymph nodes examined [21]. With the widespread use of minimally invasive gastrectomy, studies have reported similar results between the two groups regarding oncologic outcomes. However, there are different results on which of the laparoscopic and open gastrectomy methods are superior regarding lymph node count [22–26]. When robotic and laparoscopic gastrectomy were compared, a higher rate of lymph node removal was observed in the robotic gastrectomy group [27–29].

One of the best predictors of survival is lymph node status, but there are several drawbacks to the node status of TNM staging, such as being limited by the number of lymph nodes and the phenomenon of stage migration. Therefore, many studies have been conducted, and it has been found that the LNR is useful in predicting prognosis [12, 14, 30, 31].

Our study's key finding was that the ratio of metastatic lymph nodes was an independent predictor of patients' OS following curative surgery after excluding patients with multivisceral surgery, neoadjuvant treatment, and removal of 15 or fewer lymph nodes, which may affect survival.

According to Nitti et al., the ratio of metastatic lymph nodes, followed by the total number of metastatic lymph nodes (N stage in UICC), was the most important prognostic predictor among GC patients who underwent curative surgery [19]. LNR was demonstrated to be able to predict prognosis, and OS decreased with increasing LNR in both patients with more than or equal to 15 LNs investigated and those with less than 15 LNs [12]. Additionally, data from 1853 patients with GC, including those who underwent D1, D2, and D3 lymphadenectomy, were examined by Marchet et al. in 2007. Regardless of the lymphadenectomy technique and the quantity of lymph nodes that were dissected, they showed that the ratio of metastatic lymph nodes was an independent prognostic factor for patients with GC [9]. A similar large-volume study carried out in China evaluated 3864 GC patients. This study revealed that metastatic lymph node ratio (MLNR) may be a new indicator to assess the prognosis of GC patients undergoing curative gastrectomy [32].

Although the studies on this subject are generally of Far Eastern origin, there are also a few Western-centered studies [33–36]. LNR can prevent stage migration [37]. The N ratio may be used in standard clinical practice in Western countries where D1 dissection is performed, regardless of the type of lymphadenectomy. LNR would also significantly influence the selection of patients who benefit from adjuvant therapy [9, 19, 38]. However, we could not interpret this issue because our study had no adjuvant treatment data. The effect of LNR on patient selection in adjuvant treatment should be investigated in prospective studies.

Although many previous studies have reported that LNR is a more accurate prognostic factor than N stage in patients with GC, the lack of reproducibility of the threshold has made interpreting this factor problematic [13, 39, 40]. For this reason, Nakamura et al. evaluated the LNR value for each N stage and showed that combining the N stage and LNR gave better results in predicting relapse [10]. The nomograms created by combining factors such as age, sex, tumor site, and depth of invasion with LNR help to better determine the prognosis [41, 42].

Limitations of this study include the lack of disease-free survival data and the small number of patients. Prospective studies, including western and far eastern centers, may provide more enlightening information on this issue.

## Conclusions

This study showed that a high lymph node ratio was significantly associated with poor OS in patients who underwent curative gastrectomy. LNR should play a role in determining the postoperative treatment of patients and may be used as an independent prognostic predictor in GC patients.

## Data Availability

The datasets generated during and/or analyzed during the current study are available from the corresponding author on reasonable request.

## Abbreviations

GC: Gastric cancer
AJCC: American Joint Committee on Cancer
UICC: Union for International Cancer Control
TNM: Tumor-node-metastasis
LNR: Lymph node ratio
OS: Overall survival

## Declarations

Part of the data included in this manuscript has been presented as an oral presentation at the 1st International Turkish Gastric Cancer Congress, 14–16 October 2022, Izmir, Turkey, and published in Congress Abstract Book.

## References

[1] Sung H, Ferlay J, Siegel RL, Laversanne M, Soerjomataram I, Jemal A (2021). Global Cancer Statistics 2020: GLOBOCAN Estimates of Incidence and Mortality Worldwide for 36 Cancers in 185 Countries. CA Cancer J Clin.

[2] Figura N, Marano L, Moretti E, Ponzetto A (2016). Helicobacter pylori infection and gastric carcinoma: Not all the strains and patients are alike. World J Gastrointest Oncol.

[3] Joshi SS, Badgwell BD (2021). Current treatment and recent progress in gastric cancer. CA Cancer J Clin.

[4] Boccardi V, Marano L, Rossetti RRA, Rizzo MR, di Martino N, Paolisso G (2015). Serum CD26 levels in patients with gastric cancer: a novel potential diagnostic marker. BMC Cancer.

[5] Lee JY, Park MJ (2022). The Role of Serum CD26 in the Diagnosis of Gastric Cancer. Int J Gen Med.

[6] Tsai MM, Wang CS, Tsai CY, Chi HC, Tseng YH, Lin KH (2014). Potential prognostic, diagnostic and therapeutic markers for human gastric cancer. World J Gastroenterol.

[7] Zhu J, Xue Z, Zhang S, Guo X, Zhai L, Shang S (2018). Integrated analysis of the prognostic role of the lymph node ratio in node-positive gastric cancer: A meta-analysis. Int J Surg.

[8] Johnston FM, Beckman M (2019). Updates on Management of Gastric Cancer. Curr Oncol Rep.

[9] Marchet A, Mocellin S, Ambrosi A, Morgagni P, Garcea D, Marrelli D (2007). The ratio between metastatic and examined lymph nodes (N ratio) is an independent prognostic factor in gastric cancer regardless of the type of lymphadenectomy: results from an Italian multicentric study in 1853 patients. Ann Surg.

[10] Nakamura S, Kanda M, Ito S, Mochizuki Y, Teramoto H, Ishigure K (2020). Accurate Risk Stratification of Patients with Node-Positive Gastric Cancer by Lymph Node Ratio. World J Surg.

[11] In H, Solsky I, Palis B, Langdon-Embry M, Ajani J, Sano T (2017). Validation of the 8th Edition of the AJCC TNM Staging System for Gastric Cancer using the National Cancer Database. Ann Surg Oncol..

[12] Hou Y, Wang X, Chen J (2018). Prognostic significance of metastatic lymph node ratio: the lymph node ratio could be a prognostic indicator for patients with gastric cancer. World J Surg Oncol.

[13] Liu H, Deng J, Zhang R, Hao X, Jiao X, Liang H (2013). The RML of lymph node metastasis was superior to the LODDS for evaluating the prognosis of gastric cancer. Int J Surg.

[14] Wu XJ, Miao RL, Li ZY, Bu ZD, Zhang LH, Wu AW (2015). Prognostic value of metastatic lymph node ratio as an additional tool to the TNM stage system in gastric cancer. Eur J Surg Oncol.

[15] Hartgrink HH, van de Velde CJ, Putter H, Bonenkamp JJ, Klein Kranenbarg E, Songun I (2004). Extended lymph node dissection for gastric cancer: who may benefit? Final results of the randomized Dutch gastric cancer group trial. J Clin Oncol.

[16] Japanese Gastric Cancer A. Japanese gastric cancer treatment guidelines 2010 (ver. 3). Gastric Cancer. 2011;14(2):113–23. 10.1007/s10120-011-0042-4.10.1007/s10120-011-0042-421573742

[17] Seevaratnam R, Bocicariu A, Cardoso R, Yohanathan L, Dixon M, Law C (2012). How many lymph nodes should be assessed in patients with gastric cancer?. A systematic review Gastric Cancer.

[18] Marano L, D'Ignazio A, Cammillini F, Angotti R, Messina M, Marrelli D, et al. Comparison between 7th and 8th edition of AJCC TNM staging system for gastric cancer: old problems and new perspectives. Transl Gastroenterol Hepatol. 2019;4:22. 10.21037/tgh.2019.03.09.10.21037/tgh.2019.03.09PMC650942831143843

[19] Nitti D, Marchet A, Olivieri M, Ambrosi A, Mencarelli R, Belluco C (2003). Ratio between metastatic and examined lymph nodes is an independent prognostic factor after D2 resection for gastric cancer: analysis of a large European monoinstitutional experience. Ann Surg Oncol.

[20] Jian-Hui C, Shi-Rong C, Hui W, Si-le C, Jian-Bo X, Er-Tao Z (2016). Prognostic value of three different lymph node staging systems in the survival of patients with gastric cancer following D2 lymphadenectomy. Tumour Biol.

[21] Rausei S, Galli F, Lianos G, Rosa F, Cossu A, Biondi A (2020). How Should We Measure the Quality of Lymphadenectomy for Gastric Cancer? Anatomical Versus Numerical Criterion. J Gastrointest Cancer.

[22] Wei HB, Wei B, Qi CL, Chen TF, Huang Y, Zheng ZH (2011). Laparoscopic versus open gastrectomy with D2 lymph node dissection for gastric cancer: a meta-analysis. Surg Laparosc Endosc Percutan Tech.

[23] Maegawa FB, Patel AD, Serrot FJ, Patel SG, Stetler JL, Patel DC (2023). Gastric Cancer Surgery in the US: a Contemporary Trend Analysis of Lymphadenectomy and the Impact of Minimally Invasive Approaches. J Gastrointest Surg.

[24] Davey MG, Temperley HC, O'Sullivan NJ, Marcelino V, Ryan OK, Ryan ÉJ (2023). Minimally Invasive and Open Gastrectomy for Gastric Cancer: A Systematic Review and Network Meta-Analysis of Randomized Clinical Trials. Ann Surg Oncol.

[25] Lei X, Wang Y, Shan F, Li S, Jia Y, Miao R (2022). Short-and long-term outcomes of laparoscopic versus open gastrectomy in patients with gastric cancer: a systematic review and meta-analysis of randomized controlled trials. World J Surg Oncol.

[26] Marano L, D’Ignazio A, Resca L, Marrelli D, Roviello F (2021). Robotic-assisted gastrectomy for gastric cancer: single Western center results. Updates Surg.

[27] Jia Z, Cao S, Meng C, Liu X, Li Z, Tian Y (2023). Intraoperative performance and outcomes of robotic and laparoscopic total gastrectomy for gastric cancer: A high-volume center retrospective propensity score matching study. Cancer Med.

[28] Cianchi F, Indennitate G, Trallori G, Ortolani M, Paoli B, Macrì G (2016). Robotic vs laparoscopic distal gastrectomy with D2 lymphadenectomy for gastric cancer: a retrospective comparative mono-institutional study. BMC Surg.

[29] Guerrini GP, Esposito G, Magistri P, Serra V, Guidetti C, Olivieri T (2020). Robotic versus laparoscopic gastrectomy for gastric cancer: The largest meta-analysis. Int J Surg.

[30] Spolverato G, Ejaz A, Kim Y, Squires MH, Poultsides G, Fields RC (2015). Prognostic Performance of Different Lymph Node Staging Systems After Curative Intent Resection for Gastric Adenocarcinoma. Ann Surg.

[31] Persiani R, Rausei S, Biondi A, Boccia S, Cananzi F, D'Ugo D (2008). Ratio of metastatic lymph nodes: impact on staging and survival of gastric cancer. Eur J Surg Oncol.

[32] He Z, Li D, Xu Y, Wang H, Gao J, Zhang Z (2022). Prognostic significance of metastatic lymph node ratio in patients with gastric cancer after curative gastrectomy: a single-center retrospective study. Scand J Gastroenterol.

[33] Park J, Jeon CH, Kim SJ, Seo HS, Song KY, Lee HH (2021). A Novel Approach for Gastric Cancer Staging in Elderly Patients Based on the Lymph Node Ratio. J Gastric Cancer.

[34] Jiang J, Chen J, Zhang H, Rao X, Hao T, Li M, et al. Combination of the ratio between metastatic and harvested lymph nodes and negative lymph node count as a prognostic indicator in advanced gastric cancer: a retrospective cohort study. J Gastrointest Oncol. 2021;12(5):2022–34. 10.21037/jgo-21-212.10.21037/jgo-21-212PMC857625034790370

[35] Kutlu OC, Watchell M, Dissanaike S (2015). Metastatic lymph node ratio successfully predicts prognosis in western gastric cancer patients. Surg Oncol.

[36] Attaallah W, Uprak K, Gunal O, Yegen C (2016). Prognostic Impact of the Metastatic Lymph Node Ratio on Survival in Gastric Cancer. Indian J Surg Oncol.

[37] Kong SH, Lee HJ, Ahn HS, Kim JW, Kim WH, Lee KU (2012). Stage migration effect on survival in gastric cancer surgery with extended lymphadenectomy: the reappraisal of positive lymph node ratio as a proper N-staging. Ann Surg.

[38] Alatengbaolide, Lin D, Li Y, Xu H, Chen J, Wang B, et al. Lymph node ratio is an independent prognostic factor in gastric cancer after curative resection (R0) regardless of the examined number of lymph nodes. Am J Clin Oncol. 2013;36(4):325–30. 10.1097/COC.0b013e318246b4e9.10.1097/COC.0b013e318246b4e922547011

[39] Wang W, Xu DZ, Li YF, Guan YX, Sun XW, Chen YB, et al. Tumor-ratio-metastasis staging system as an alternative to the 7th edition UICC TNM system in gastric cancer after D2 resection--results of a single-institution study of 1343 Chinese patients. Ann Oncol. 2011;22(9):2049–56. 10.1093/annonc/mdq716.10.1093/annonc/mdq71621310759

[40] Alakus H, Kaya M, Mollaoglu MC, Göksu M, Ozer H, Karadayi K. Negative-to-Positive Lymph Node Ratio as an Independent Prognostic Factor for Gastric Adenocarcinoma. Journal of the College of Physicians and Surgeons--Pakistan : JCPSP. 2021;30(7):805–10. 10.29271/jcpsp.2021.07.805.10.29271/jcpsp.2021.07.80534271780

[41] Kim Y, Spolverato G, Ejaz A, Squires MH, Poultsides G, Fields RC (2015). A nomogram to predict overall survival and disease-free survival after curative resection of gastric adenocarcinoma. Ann Surg Oncol.

[42] Capelli G, Tonello AS, Chiminazzo V, Lorenzoni G, Bao QR, Marchet A (2022). Validation of a Nomogram to Predict Long Term Outcomes After Curative Surgery for Gastric Cancer in an Italian Cohort of Patients. J Visc Surg.

